# Phytochemical Profile and Antioxidant and Antiproliferative Activity of *Sedum dendroideum* on Pterygium Fibroblasts

**DOI:** 10.1155/2021/5814221

**Published:** 2021-10-18

**Authors:** Paloma López-Montemayor, Judith Zavala, María Dolores Montalvo-Parra, Guillermo Isaac Guerrero-Ramírez, Karla Mayolo-Deloisa, Daniela Enriquez-Ochoa, Bernardo Martínez-García, Denise Loya-García, Alba Miriam Guerrero-Martínez, Jorge Eugenio Valdez-García

**Affiliations:** ^1^Tecnologico de Monterrey, Escuela de Medicina, 3000 Morones Prieto Ave, Col. Los Doctores, C. P. 64710, Monterrey, Nuevo Leon, Mexico; ^2^Tecnologico de Monterrey, Escuela de Ingenieria y Ciencias, 2501 Eugenio Garza Sada Ave, Col. Tecnologico, C. P. 64849, Monterrey, Nuevo Leon, Mexico

## Abstract

**Background:**

*Sedum dendroideum* has antioxidant effects that are beneficial for different diseases. We aimed to analyze the antiproliferative activity of *S. dendroideum* in human pterygium fibroblasts (HPFs).

**Methods:**

HPFs were treated for 24 h with 0–1000 *μ*g/mL of *S. dendroideum* lyophilized to analyze its effect on cell viability using the CellTiter assay. RNA from HPF treated with 250 *μ*g/mL of *S. dendroideum* lyophilized was isolated, and the expression of VEGF and CTGF genes was evaluated by qPCR. A dermal fibroblast cell line (HDFa) was used as a healthy control. The total phenolic content, antioxidant activity, and chemical profile of *S. dendroideum* lyophilized were determined.

**Results:**

Viability of HPF decreased after 24 h treatment of *S. dendroideum* in a dose-dependent manner. The expression of VEGF and CTGF significantly decreased (*P* < 0.01) in HPF treated with 250 *μ*g/mL of *S. dendroideum* when compared with untreated HPF. The total phenolic concentration in the *S. dendroideum* lyophilized was 33.67 mg gallic acid equivalents (GAE)/g. Antioxidant activity was 384.49 mM Trolox equivalents/mL. The main phenolic compounds identified by HPLC analysis were the kaempferol-3-O-glycoside, kaempferol-3-O-rhamnoside, kaempferol-3-O-neohesperidoside-7-O-*α*-rhamnopyranoside, and kaempferol-3-O-glycoside-7-O-rhamnoside.

**Conclusions:**

*S. dendroideum* decreases the proliferation of HPF and the expression of VEGF and CTGF. The phenolic compound concentration, antioxidant activity, and phytochemical profile may play a role in these effects.

## 1. Introduction

Succulent plants, or Sempervivum, are part of the Crassulaceae family and are well known for their medicinal properties. The *Sedum* genre has more than 30 species. *S. dendroideum* is a species commonly used in Brazilian and Mexican traditional medicine due to its analgesic, antimicrobial, and gastroprotective properties. Previous scientific reports proved its activity against pain (antinociceptive) in an induced peritonitis model, antioxidant activity used as a fresh leaf infusion, antiglycemic effect in diabetic mice, anti-inflammatory activity *in vitro* due to its ability to stimulate macrophages to produce cytokines, and gastroprotective effect *in vivo* [1–4]. These properties are related to vegetal secondary metabolites, including flavonoids glycosides, tannins, kaempferol, quercetin, and phenols. Given the potential of *S. dendroideum*, we aimed to analyze it for a common ocular disease for which there is no pharmacological treatment. Pterygium is a wing-shaped tissue growth over the conjunctiva. It produces ocular irritation, foreign body sensation, and prurience, and its growth can interfere with the visual field [5]. It has tumor-like characteristics such as growth, migration, inflammation, and neovascularization. However, it is considered a benign growth because it does not metastasize. Pterygium prevalence is up to ∼10% within the population of areas at a high risk considering the mean annual UV index, such as regions near the equator [6]. The only treatment available is surgical removal, with a variable recurrence rate [7]. Pterygium pathogenesis is not fully understood; however, long-term sun ultraviolet-B (UV-B) radiation exposure and environmental pollution are well-documented risk factors. This leads to dysregulation of molecules such as interleukins 1, 6, and 8; the growth factors VEGF, PDGF, bFGF, and CTGF; and metalloproteinases involved with the processes of inflammation, cell migration, proliferation, oxidative stress, and neovascularization [8, 9]. These cellular processes could be mitigated by the proven activity of *S. dendroideum*. Dysregulation of these molecular processes has been reported for both cell types of pterygium, epithelium, and fibroblasts.

Given the molecular properties proven of *S. dendroideum*, we aimed to analyze its effect on human pterygium fibroblasts by means of proliferation along with the chemical profile of possible active compounds. Thus, this provides evidence for the development of a potential pharmacological treatment for pterygium.

## 2. Materials and Methods

### 2.1. Plant Materials and Sap Extraction

The *S. dendroideum* plant was collected from a vivarium in Santiago, Nuevo Leon, Mexico. The stems and leaves (176.04 g) were blended with 100 mL of distilled H_2_O, filtrated, and frozen at −80°C for 24 h. The solution was lyophilized for 6 days with a yield of 3.979 g. A stock solution of 100 mg of lyophilized powder in 1 mL of DMSO (Sigma-Aldrich, Missouri, USA) was prepared, filtered with a 0.22 *μ*M filter (Corning, New York, USA), and stored at −20°C.

### 2.2. Human Pterygium Fibroblast Primary Culture

The study was conducted in accordance with the Declaration of Helsinki. Four surgically removed pterygiums were donated by Hospital La Carlota, Montemorelos, NL. A small fraction (3 mm approximately) of each pterygium was fragmented and cultured with DMEM-F12 (Gibco, New York, USA) supplemented with 5% SBF and 1% antibiotic at 37°C in a humidified chamber with 5% CO_2_. The medium was changed every third day upon confluence. Tissue fragments were removed from culture plates before the first passage. All cells were used from passage 3 to 10 for experimentation. As healthy control, a cell line (ATCC®PCS-201-012) of human dermal fibroblast (HDFa) was used.

### 2.3. Characterization of Pterygium Fibroblasts

To characterize the pterygium fibroblasts isolated from primary culture, the expression of keratin, Aldh3, and Prdx2 was analyzed by immunofluorescence. HPFs were fixed using 4% paraformaldehyde and stained for Aldh3a1 (1 : 100), Prdx2 (1 : 500), and pan-keratin (1 : 10) (Abcam, Cambridge, MA). Images were taken with a structured illumination microscope (Zeiss ApoTome-DZNE W1).

### 2.4. Cell Viability Assay

Dilutions of the lyophilized stock solution were prepared using DMEM-F12 sterilized media. HFDa and HPF were treated with 0, 250, 500, 1000, and 1500 *μ*g/mL of *S. dendroideum* for 24 h. Each dose was tested in triplicate. Cell viability was analyzed with the CellTiter-Blue Cell Viability Assay (Promega, Wisconsin, USA) according to the instructions provided by the manufacturer. In brief, cells were plated in 96-well culture plates at a density of 5000 cells per well in 200 *μ*L of medium and incubated overnight. The medium was replaced with medium (200 *μ*L/well) containing different concentrations of *S. dendroideum*. After 24 h, the medium was replaced with medium supplemented with the CellTiter-Blue reagent. After incubation for 1 h, the fluorescence of the medium was measured using the Synergy HT Multi-Detection Microplate Reader. Pilot experiments indicated that seeding 5000 cells/well and incubating the cells with CellTiter-Blue reagent for 1 h after *S. dendroideum* treatment were optimal conditions.

### 2.5. VEGF and CTGF Expression Analysis

To evaluate the effect of *S. dendroideum* sap over the expression of CTGF and VEGF, a concentration of 250 *μ*g/mL was used. This concentration was obtained as the half-maximal inhibitory concentration (IC50) in preliminary analysis (data not shown). Total RNA of HFDa and HPF treated with 250 *μ*g/mL of *S. dendroideum* sap and from untreated HPF was isolated using Trizol reagent according to the manufacturer's instructions (Merck, Darmstadt, Germany). cDNA was generated from RNA using the High-Capacity cDNA Reverse Transcription Kit (Applied Biosystems, California, USA). Each reaction contained 2 *μ*L of buffer 10X, 0.8 *μ*L of dNTPs, 2 *μ*L of random primers, 1 *μ*L of RT enzyme, and 4.2 *μ*L of nuclease-free water. The thermal cycler was run using the following program: primer annealing for 10 min at 25°C, reverse transcription for 120 min at 37°C, and enzyme deactivation for 5 min at 85°C. The qPCR was carried out using PowerUp Green Master Mix (Applied Biosystems). Each sample contained 10 *μ*L of SYBR Green, 7.4 *μ*L of nuclease-free water, 0.6 *μ*L of primer, and 2 *μ*L of cDNA. Primer sequences used (Integrated DNA Technologies) are shown in Table 1. To calculate the level of mRNA relative expression, values were analyzed using ΔΔCt using GAPDH as the endogenous gene.

### 2.6. *S. dendroideum* Phenolic Concentration Analysis

The total phenolic content was determined by means of spectrophotometric analysis with the Folin–Ciocalteu method. The concentration of polyphenols was quantified through a calibration curve of gallic acid equivalents (mg/mL). Folin–Ciocalteu reactive (Sigma-Aldrich) was used to analyze the dilutions of *S. dendroideum* samples. The results were expressed as gallic acid equivalents (mgGAE/mg dry lyophilized). This analysis was performed in triplicate.

### 2.7. *S. dendroideum* Antioxidant Activity

An oxygen radical absorbance capacity (ORAC) assay in 96-well multidetection plates was determined. Fluorescence sodium (Sigma, St. Louis, MO, USA) was used as a fluorescence probe, Trolox as a standard free radical scavenger, and AAPH as the peroxyl radical generator.

For 1 hour, the fluorescence was measured in a Synergy HT Multi-Detection Microplate Reader at 37°C with excitation/emission at 485/528 nm every 2 minutes.

### 2.8. HPLC Phenolic Compounds Analysis

The phenolic compound profile of *S. dendroideum* extract was evaluated on a 1260 Infinity HPLC system coupled to a diode array detector (DAD) (Agilent Technologies, CA, USA). The HPLC method followed has been reported previously [10]. In brief, the analysis was developed using a 5 *μ*m Luna C18 reverse-phase column (Phenomenex, CA, USA), maintained at 25°C. The mobile phase consisted of water (eluent A) and methanol-water (60 : 40% v/v, eluent B). The pH of both eluents was adjusted to 2.4 using phosphoric acid (D. E. Q., Monterrey, NL, Mexico). The gradient used was as follows: 0 min, 100/0; 3 min, 70/30; 8 min, 50/50; 35 min, 30/70; 40 min, 20/80; 45 min, 0/100; 50 min, 0/100; and 60 min, 100/0 (time (%) of eluent A/% of eluent B). The method was run for 60 min at 0.8 mL/min with a pressure of no more than 400 psi. The samples were prepared in DMSO (Research Organics, Cleveland, OH, USA) and further diluted with water to a final concentration of 25 mg/mL. Chromatograms were recorded at 360 nm.

## 3. Results

### 3.1. The Influence of *S. dendroideum* on HPFs

Cultured HPFs expressed Aldh3, Prdx2, and pan-keratin (Figure 1) when analyzed by immunocytochemistry.

The reduction in cell viability after 24 hours of treatment was dose dependent. The IC50 was 208 *μ*g/mL. The viability of HFDa did not decrease with the treatment of *S. dendroideum* (Figure 2(a)).

The gene expression of VEGF and CTGF showed a significant decrease (*P* < 0.01) in HPF treated with 250 *μ*g/mL of *S. dendroideum* lyophilized sap compared with untreated cells. HFDa did not show a decrease in VEGF or CTGF expression after *S. dendroideum* lyophilized sap treatment (Figures 2(b) and 2(c)).

### 3.2. Characterization of *S. dendroideum*

The antioxidant activity of *S. dendroideum* analyzed by the AAPH method was 384.49 mM Trolox equivalents/mL. The total polyphenol content of *S. dendroideum* dry lyophilizate was determined by the method of Folin–Ciocalteu assay, thus obtaining 33.67 mg gallic acid equivalents (GAE)/g. The HPLC profile of *S. dendroideum* showed several peaks corresponding to different phenolic compounds (Figure 3).

The retention time, maximum absorbance, and the percentage area of the main peaks are observed in Table 2. To get a better insight into *S. dendroideum* chemical composition, the peaks were tentatively identified by comparing their UV spectrum and retention time with available data reported in the literature. The results suggest that the main phenolic compounds in *S. dendroideum* are kaempferol glycosides, such as kaempferol-3-O-glycoside, kaempferol-3-O-rhamnoside, kaempferol-3-O-neohesperidoside-7-O-*α*-rhamnopyranoside, and kaempferol-3-O-glycoside-7-O-rhamnoside.

## 4. Discussion

Pterygium is a disease with a high prevalence in regions near to the equator. It affects people whose activities involve chronic exposure to UV radiation. The only treatment available is surgical removal, which is not completely effective and may not be economically accessible to the main population affected. Several studies on *S. dendroideum* have found it to be beneficial in inflammatory and chronic diseases [1, 3, 11]. We aimed to analyze the activity of *S. dendroideum* over pterygium fibroblasts.

Pterygium fibroblasts have dysregulation in several molecular pathways related to antioxidant activity, migration, inflammation, and proliferation [8, 12]. Some of these molecules are upregulated in pterygium samples, including ALDH3 and PRDX2. The former acts as a defense against UV-induced oxidative stress on the ocular surface [13], while PRDX2 contributes as part of the antioxidant defense by inactivating hydrogen peroxide [14]. Specific forms of keratin, including keratin 13 and 4, are increased in pterygium and have a role in cell migration [15]. These three biomarkers were detected in the primary isolated HPF of this work.

HPFs treated with *S. dendroideum* lyophilized sap showed a dose-dependent viability decrease, while HFDa remained viable at all dosages. These results are in accordance with previous studies that demonstrated the antiproliferative effect of extracts from plants from the same family. A crude whole plant fraction from *S. sarmentosum* inhibits the growth of hepatocellular carcinoma and of a pancreatic cell line in a dose-dependent manner [16, 17]. For pterygium treatment, there are reports showing promising efficacy of plant-derived extracts. In a study conducted with 13 patients having pterygium or pinguecula treated with an herbal formulation, a 76.9% response improvement was registered [18]. The cited study did not describe how the improvement was assessed, and none of the herbal components were from the succulent variety nor chemically characterized. Similar studies report mild anti-inflammatory activity of *Physalis peruviana* and *Curcuma longa* extracts over a rabbit pterygium model and cultured pterygium keratinocytes, respectively [19, 20]. The inhibition of pterygium keratinocytes in the mentioned study was related to an increase in apoptotic activity. In our study, VEGF and CTFG expression changes were assessed. VEGF is an angiogenic cytokine with a pivotal role in normal and pathological angiogenesis and is upregulated in pterygium after UV radiation [21]. CTGF promotes connective tissue remodeling, thus activating tissue migration in pterygium [22]. Although the expression of these molecules has been reported as possible therapeutic targets, there is a lack of studies showing the effect of herbal extract treatment on these cytokines in pterygium. In our study, the expression of VEGF and CTGF was decreased after *S. dendroideum* treatment. This effect was not seen in healthy dermal fibroblasts. Recent studies report the arrest in pterygium proliferation with a decrease of VEGF using 5-fluorouracil (5FU) injection, an antifibrotic agent that inhibits the synthesis of DNA [23, 24]. However, this treatment may produce hyperemia, keratitis, and pain and will not be entirely effective in preventing recurrence [25]. Further studies are needed to analyze the ability of *S. dendroideum* components to decrease VEGF and other pterygium cytokines with no side effects. The combination of the phytochemical compounds found in *S. dendroideum* could help in exerting beneficial activity without unwanted secondary effects. *S. dendroideum* had higher antioxidant activity (384.49 mM Trolox equivalents/mL) and total phenolic content (33.67 mg gallic acid equivalents (GAE)/g) than other plants in the Crassulaceae family, including *Umbilicus intermedius*, *Umbilicus rupestris*, and *Sedum sempervivoides* [26]. *S. dendroideum* phenolic content is within the average of that reported in other *Sedum* species, such as *S. maximum* and *S. acre* [27, 28]. The compound profile found by HPLC analysis is consistent with previous reports, in which kaempferol glycosides have been identified as the most abundant compounds in *S. dendroideum* leaf juice and freeze-dried leaves [2, 11, 29]. The analysis of *S. dendroideum* freeze-dried leaves also showed the presence of myricetin and quercetin glycosides [2]. Furthermore, kaempferol, myricetin, and quercetin glycosides have been reported in species from the Crassulaceae family [30–35]. Myricetin, quercetin, and kaempferol aglycone from *S. dendroideum* have been linked to antioxidant, anti-inflammatory, antinociceptive, and gastroprotective activity [1, 2, 4, 11].

## 5. Conclusions

*S. dendroideum* is a plant well known for its healing properties in traditional medicine. In the ophthalmological area, there is a need for the pharmacological treatment of diseases of the ocular surface, such as pterygium. *S. dendroideum* showed activity in the decrease of the proliferation of HPF and the expression of VEGF and CTGF. The phenolic compound concentration, antioxidant activity, and phytochemical profile may play a role in these effects. These results set the baseline for further studies *in vivo* to test the preventive or therapeutic activity of *S. dendroideum.*

## Figures and Tables

**Figure 1:** Immunodetection of Aldh3, keratin, and Prdx2 in primary isolated pterygium fibroblasts.

**Figure 2:** Cell viability changes of HPF and HFDa after treatment with *S. dendroideum* lyophilized (a). A significant decrease when analyzed with a *t*-test (*P* < 0.01) is registered in the expression of VEGF (b) and CTGF (c) in HPF treated with 250 *μ*g/mL of *S. dendroideum* lyophilized compared with untreated cells (control).

**Figure 3:** Phenolic compounds' profile in *S. dendroideum* obtained by HPLC-DAD at 360 nm.

**Table 1:** Primer sequences for different genes. The sequences are listed in the 5′–3′ direction.

Gene	F_Primer	R_Primer
VEGF	TGGTTCCCGAAACGCTGAG	TGCCCACTGAGGAGTCCAAC
CTGF	GAAGGGCAAAAAGTGCATCC	GAAGGGCAAAAAGTGCATCC
GAPDH	GAGTCAACGGATTTGGTCGT	TTGATTTTGGAGGGATCTCG

**Table 2:** Retention time (*t*_R_), maximum absorption wavelengths (*λ*_max_), and percentage area (%) from the main peaks of phenolic compounds' profile obtained using HPLC-DAD at 360 nm.

Peak number	*t*_R_ (minutes)	*λ*_max_ (nm)	Tentative identification	%
1	15.283	Not determined	Not identified	1.4320
2	18.708	Not determined	Not identified	2.4539
3	21.719	272, 334	Apigenin-7-O-glycoside^a^	4.0420
4	25.021	254 sh, 264, 296 sh, 316 sh, 354	Kaempferol-3-O-glycoside^a^	8.9907
5	26.154	246 sh, 268, 318 sh, 348	Kaempferol-3-O-glycoside-7-O-rhamnoside^a^	5.2386
6	27.864	246 sh, 266, 318 sh, 348	Kaempferol diglycoside^a^	4.2962
7	30.504	246 sh, 266, 320 sh, 348	Kaempferol diglycoside^a^	3.7200
8	31.976	Not determined	Not identified	4.6247
9	38.552	224 sh, 264, 322 sh, 348	Kaempferol glycoside^b^	21.9344
10	44.533	266, 298 sh, 356	Kaempferol-3-O-rhamnoside^c^	14.7406
11	45.271	228 sh, 264, 314 sh, 344	Kaempferol-3-O-neohesperidoside-7-O-*α*-rhamnopyranoside^d^	17.0646

sh, shoulder. Identification based on the data reported by [10]^a^, [11]^b^, [12]^c^, and [30]^d^.

## Data Availability

The data used to support the findings of this study are available from the corresponding author upon request.
